# S100A8/A9 Molecular Complexes Promote Cancer Migration and Invasion via the p38 MAPK Pathway in Nasopharyngeal Carcinoma

This article has been retracted.

**DOI:** 10.1155/2021/9913794

**Published:** 2021-06-22

**Authors:** Ning Xu, Bei-Bei Zhang, Xia-Ning Huang, Xiang Yi, Xue-Min Yan, Yan Cai, Qin He, Zi-Jian Han, Yuan-Jiao Huang, Wei Liu, Ai-Jun Jiao

**Affiliations:** ^1^The Fifth Affiliated Hospital of Guangxi Medical University, Nanning, China; ^2^Institute of Biomedical Research, Yunnan University, Kunming, China; ^3^Wuming Hospital of Guangxi Mediacal University, Nanning, China; ^4^Department of Otolaryngology-Head and Neck Surgery, The First Affiliated Hospital of Guangxi Medical University, Nanning, China; ^5^Graduate School of Guangxi Medical University, Nanning, China; ^6^Life Science Institute, Guangxi Medical University, Nanning, China; ^7^School of Basic Medical Sciences, Guangxi Medical University, Nanning, China; ^8^Pharmaceutical College, Guangxi Medical University, Nanning, China

## Abstract

Nasopharyngeal carcinoma (NPC) is one type of malignancy associated with migration and invasion through a currently unclear mechanism. We previously discovered S100A8/A9 levels were roughly elevated in the plasma of NPC patients as the promising biomarkers. However, their expressions and underlying functions in NPC tissues are still unknown. In the present study, we analyzed 49 NPC tissues and 20 chronic pharyngitis (CP) tissues. Immunohistochemical staining was performed in different tissues and analyzed by the Mann–Whitney *U* test statistically. Transwell migration and invasion experiments were further performed to determine S100A8/A9 effects on NPC. Our results showed that S100A8/A9 in NPC tissues were significantly higher than those in CP tissues, closely associated with NPC clinical stages. Intriguingly, exogenous S100A8/A9 protein stimulation could dramatically enhance NPC migration and invasion abilities. In addition, p38 MAPK pathway blockade could diminish the migration and invasion of NPC cells stimulated by S100A8/A9 proteins. The downstream tumor invasion and migration associated proteins (e.g., MMP7) were also elevated in NPC tissues, consistent with S100A8/A9 overexpression. Taken together, our present findings suggest that the secreted soluble inflammatory factors S100A8/A9 might promote cancer migration and invasion via the p38 MAPK signaling pathway along with invasion/migration associated proteins overexpression in the tumor microenvironment of NPC. This may shed light on the mechanism understanding of NPC prognosis and provide more novel clues for NPC diagnosis and therapy.

## 1. Introduction

Nasopharyngeal carcinoma (NPC) is the most common otorhinolaryngological tumor type originated from the epithelial cells [1, 2]. In 2018, the new incidence was estimated as 130,000 cases from the latest global cancer surveillance report [3]. NPC is well known as a cancer type characterized by distinct ethnic and regional specificity [4]. Endemic to China, this malignancy represents a variable occurrence rate ranging from the high incidence (southern China) to a low rate (northern China), while it is a rare disease among Caucasians [4]. Southern China (e.g., Guangdong and Guangxi) suffers a very high-risk of NPC, where the incidence ratio is much higher than the world's [5, 6]. Nonkeratinized low differentiation NPC with high degree of malignancy is the main pathological type in clinical [7]. As high as 60–70% of the newly diagnosed NPC patients have already developed local advanced lesions [8, 9]. Along with the development of modern radiotherapy and chemotherapy, the initial treatment response rate currently reaches 90.9% for these NPC patients with advanced stages (III and IV stages) [10], and the five-year survival rate is 72.3–86% [11–13]. However, NPC often has a high incidence of recurrence and distant metastasis, especially for those patients with advanced stages. As for them, the five-year incidence is 20–30% [14, 15] and the ten-year incidence is 30–40% [16]. What is worse, the treatment response rate decreases to 65.8–66.7% [17, 18] and median survival time is just 14.0–27.2 months [17, 19]. These biological characteristics and the abundant peripheral lymphoid tissue involvement make NPC more prone to the metastasis and invasion compared with the other head and neck tumor types. The recurrence and distant metastasis are causes of treatment failure for NPC patients. Consequently, the majority of patients succumb to the effects of tumor metastasis rather than to the primary lesion. To better promote NPC prognosis and provide a rationale for novel therapies, it was absolutely essential to discover more promising biomarkers of NPC and unravel their underlying molecular mechanisms.

We previously developed a high-flux proteomic classification system to provide the highly accurate and innovative approach for NPC detection and diagnosis [20]. In the recent study, the plasma proteins from 244 NPC patients (II stage: 36 cases; III stage: 104 cases; IV stage: 104 cases) and 104 healthy donors were screened to discover potential novel NPC biomarkers using the techniques of isobaric tags for relative and absolute quantitation (iTRAQ) and liquid chromatography tandem mass spectrometry (LC-MS/MS). These NPC patients did not receive any treatment before diagnosis and were excluded if they had infection, diabetes, hypertension, autoimmune inflammation, and other diseases. The findings showed that both of the S100A8 and S100A9 protein levels in the plasma of these NPC patients diagnosed at any different clinical stages were obviously higher than those in healthy donors, which suggested that S100A8/A9 may be the potential plasma biomarkers for NPC diagnosis [21].

S100A8 (calgranulin A, MRP8) and S100A9 (calgranulin B, MRP14) are a pair of calcium binding proteins in S100 protein family, which often form a heterodimer complex in a calcium-dependent manner. They have the amino terminal ef-1 and carboxyl terminal ef-2 hand domains with low molecular weight (Mr 14000 and 13000, respectively) and display important functions in immunity [22, 23]. Tumor microenvironment (TME) is closely related to tumor occurrence and metastasis. The interactions between soluble factors in microenvironment and tumor cells play important roles in cancer development [24–27]. S100A8/A9 is a pair of secreted soluble inflammatory factors. Their main function is to drive a strong chemotaxis effect on the aggregation, adhesion, and migration of white blood cells, as well as amplify the local inflammatory effects in microenvironment [28, 29]. To date, the expression of S100A8/A9 proteins in tumor tissues and their roles in microenvironment is still unknown for NPC.

In this study, we would uncover the expression status of S100A8 and S100A9 proteins in NPC tissues and further reveal a molecular basis for their effects on NPC cell proliferation, migration, and invasion, which might provide a rationale for NPC prognosis and novel treatment.

## 2. Materials and Methods

### 2.1. Paraffin Tissue Samples

Paraffin embedded tissue samples with detailed pathological diagnosis information were collected from the Pathology Department of the Affiliated First Hospital, Guangxi Medical University, from January 2013 to June 2014, and the Pathology Department of the Affiliated Cancer Hospital, Guangxi Medical University, from March 2012 to April 2013. Through careful inquiry of medical record information, only these NPC samples were included considered that the patients have not received any radiotherapy, chemotherapy, or targeted therapy before diagnosis and have no interference of other diseases including infection, hypertension, diabetes, or autoimmune inflammation. Professional pathologists confirmed the NPC tissues were nonkeratinizing undifferentiated carcinoma, and the degree of tissue infiltration (TI), lymph node metastasis (LNM) and clinical stage (CS) were based on the criteria of the Union for International Cancer Control (UICC, 8th Edition). The structure of NPC tissue samples was clear. The relevant study was conducted in accordance with the Declaration of Helsinki, and the protocol was approved by the patients' informed consents and the Medical Ethics Committee of Guangxi Medical University (No. 050312).

### 2.2. Cell Culture and Cell Proliferation

Human NPC cell lines CNE1 (high differentiation), CNE2 (low differentiation), and 6-10B (tumorigenesis and low metastasis) were all purchased from Cell Bank of Xiangya Central Laboratory, Hunan province, China. All the cell lines were cultured in RPMI 1640 medium (HyClone Company, USA) supplemented with 10% fetal bovine serum (Gibco Company, US), penicillin, and streptomycin at 37°C, 5% CO_2_. The CCK8 assay was performed to test the cell proliferation, according to the manufacturer's instructions.

### 2.3. S100A8/A9 Solution Preparation

The S100A8 recombinant protein (Human, Amresco, USA) and S100A9 recombinant protein (Human, Amresco, USA) were mixed in a 1 : 1 ratio and placed at 4°C for 1 h to form the complex (S100A8/A9).

### 2.4. Immunohistochemistry

The expression levels of S100A8 and S100A9 in NPC tissues and CP tissues were detected by immunohistochemistry (IHC). Tissue sections (6 *μ*m) were used for dewaxing, hydration, and antigen repair. S100A8 monoclonal antibody (1 : 250, rabbit, Abcam, USA) and S100A9 monoclonal antibody (1 : 350, rabbit, Abcam, USA) were used for the primary antibody incubation; PV-9000 reagent was used for secondary antibody incubation (Beijing Zhongshanjinqiao Company, China); DAB solution was used for color rendering (Beijing Zhongshanjinqiao Company, China). After section preparation, an inverted microscope (Olympus, Japan) was used for sample observation. Five fields (200×) were taken from the top, bottom, left, right, and middle, respectively, for each sample slide. The software of Cell Sens Dimension was used to identify positive staining color (brown-yellow or tan) and calculate the percentage of positive staining cells in each field of vision. The positive imaging sample provided by the reagent provider was used as the positive control, and PBS instead of primary antibody was used as the negative control. Similarly, rabbit *β*-catenin monoclonal antibody (Abcam, USA) and rabbit MMP7 polyclonal antibody (OriGene, USA) were also used for the protein detection in clinical tissues.

### 2.5. Transwell Migration and Invasion Experiment

The effect of S100A8/A9 on the migration ability of NPC cells was tested by transwell migration assay. CNE1, CNE2, and 6-10B cells in the logarithmic growth phase were cultured for 12 h for serum starvation and then seeded into the upper chamber of transwell (1×10^5^cells/well). RPMI 1640 medium containing 10% fetal bovine serum and 1 *μ*g/ml S100A8/A9 was added in the lower chamber of transwell as the experimental group. A control group without S100A8/A9 protein was set for each cell line. After culture for 24 h, five fields (200×, top, bottom, left, right, and middle, respectively) on the down surface of the polycarbonate membrane were photographed using the inverted microscope (Olympus, Japan). The cells were counted, and the average value was taken for statistics.

The effect of S100A8/A9 on the invasion ability of NPC cells was tested by transwell invasion assay. Matrigel was diluted with precooled RPMI 1640 medium at the ratio of 1 : 6, and 100 *μ*l mixture was evenly spread on the bottom of the upper chamber of the transwell chamber to prepare the coating of basement membrane; subsequently, the basement membrane was rehydrated using medium. The following steps are the same as the transwell migration experiment above. Similarly, 1 *μ*g/ml S100A8/A9 was added to the lower chamber culture medium for the experimental group, while those without S100A8/A9 were set as the control groups.

### 2.6. Inhibition Experiment of the p38 MAPK Pathway and MEK Pathway

Transwell assay was carried out after p38 MAPK pathway blockade using SB203580 to examine the effect of S100A8/A9 on NPC cell migration and invasion. SB203580 (CST, USA) dissolved in DMSO (Amresco, USA) was used to make 10 *μ*M working concentration. Cells in the logarithmic growth phase were cultured for 12 h for serum starvation and then divided into two groups. Experimental group: cells pretreated with SB203580 for 1 h and were cultured in RPMI 1640 medium containing 10% fetal bovine serum and 1 *μ*g/ml S100A8/A9. Control group: cells pretreated with the same amount of DMSO as in the experimental group and cultured in RPMI 1640 medium containing 10% fetal bovine serum and 1 *μ*g/ml S100A8/A9. Transwell migration and invasion experiments were carried out according to the experimental methods above. As for the MEK pathway blockade, the MEK1/2 selective inhibitor AZD6244 compound (CST, USA) was used, and the similar experiments were performed.

### 2.7. Statistics

All experimental data were statistically processed using SPSS 16.0 software. The area percentage of S100A8 and S100A9 positive staining cells was tested by normality and homogeneity of variance. They did not conform to the normal distribution, and the variances were not homogeneous. Therefore, the nonparametric statistical method was used. The comparisons between different groups were analyzed by the Mann–Whitney *U* test. In the transwell migration and invasion experiment, these measurement data were shown as mean plus or minus standard deviation. These experimental results conform to the normal distribution. Student's *t*-test was used for statistical analysis between different groups. Three independent experiments were repeated for each assay. The *P* value less than 0.05 was considered statistically significant for all the experiments.

## 3. Results

### 3.1. S100A8 and S100A9 Proteins Were Frequently Overexpressed in Clinical NPC Tissues

To clarify the expression status of S100A8 and S100A9 proteins in NPC tissues, we performed the immunohistochemistry experiments to observe their expressions in 49 NPC cases and 20 chronic pharyngitis (CP) cases. Interestingly, we found a large number of brown-yellow staining signals for S100A8 proteins in the intercellular space and tumor cell cytoplasm of these NPC tissues including phases II, III, and IV, while there was only a few brown-yellow staining in CP tissues (Figures 1(a) and 1(b)). Similarly, a large number of brown-yellow staining signals for S100A9 proteins were also detected in the intercellular space and tumor cell cytoplasm of these NPC tissues including phases II, III and IV, while only a few brown-yellow staining for S100A9 was observed in CP tissues (Figures 1(c) and 1(d)). The results indicated that abundant S100A8 and S100A9 proteins were expressed in NPC tissues including II, III and IV clinical stages, mainly distributed in the columnar epithelial interstitium and in the cytoplasm of NPC cells. In contrast, only a few S100A8 and S100A9 proteins existed in the CP tissues, and most of them were concentrated in the columnar epithelial interstitium of tissues.

The statistically analyzed results showed that the positive staining area percentage (PSAP) of S100A8 and S100A9 in 49 cases of NPC tissues was 11.74 (8.08, 22.91) and 14.97 (10.55, 21.40), respectively, which were higher than those of 0.29 (0.07, 1.39) and 3.21(1.98, 3.89) in 20 cases of CP tissues, with the significant differences (*z* values −6.34 and −5.95, *P* < 0.01, respectively) (Figures 1(b) and 1(d) and Table S1).

### 3.2. S100A8 and S100A9 Expression Levels Were Closely Related to NPC Clinical Stages

In further stratified analysis, positive stained area percentages of S100A8 and S100A9 in II, III, or IV stage NPC tissues were both significantly higher than CP tissues (*P* < 0.01, respectively) (Figures 1(b) and 1(d) and Table S2). In addition, the positive staining area percentages of S100A8 and S100A9 in advanced stage NPC (III stage or IV stage) were significantly higher than those in early stage NPC (II stage) (*P* < 0.01, respectively) (Table S2), while the III stage and IV stage were not statistically different (Figures 1(b) and 1(d) and Table S2).

Importantly, we also explored the correlation between positive staining area percentage of S100A8 and S100A9 in NPC tissues and clinical features. Our data suggested that the expression levels of S100A8 and S100A9 in NPC tissues were not related to sex and age, tissue invasion, and lymphatic node metastasis, but closely related to the clinical stage (*P* < 0.05, respectively) (Table S3).

### 3.3. S100A8/A9 Stimulation Promotes NPC Cell Proliferation, Migration, and Invasion

We previously found S100A8/A9 proteins were overexpressed in NPC cells, and silencing of endogenous S100A8/A9 could significantly reduce NPC cell migration ability [30]. S100A8/A9 as a pair of secreted soluble inflammatory factors was also detected in the intercellular space besides the tumor cell cytoplasm in these NPC tissues as indicated above. To explore the effects of exogenous S100A8/A9 on NPC cell proliferation, we treated the NPC cells with S100A8/A9 at different concentrations to mimic S100A8/A9 infiltrated NPC microenvironment and detected cell proliferation by CCK8 assay. The results suggest that all the three cell lines of CNE1 (high differentiation), CNE2 (low differentiation), and 6-10B (low tumorigenesis and metastasis) have already tended to increase their growths significantly in a dose-dependent manner with S100A8/A9 treatment for 24 h, although there is still no overwhelming change in cell proliferation within the range of 0–5 *μ*g/ml S100A8/A9 concentrations we tested (Supplementary Figure S1).

In addition to the cancer cell proliferation, migration, and invasion, underlying metastatic dissemination is the key clinical problem in NPC. The present clinical investigation indicated NPC prognosis was remarkably associated with S100A8/A9 protein expression abundances. To further explore the effects of S100A8/A9 protein stimulation on NPC migration and invasion, we carried out the transwell migration and invasion experiments using these NPC cell culture models. Interestingly, the results indicated that as low as 1 *μ*g/ml S100A8/A9 added to the lower chamber culture medium could already significantly drive the migration and invasion towards S100A8/A9 stimulation for all the three NPC cell lines including CNE1, CNE2, and 6-10B (Figures 2(a)–2(c)). Moreover, we predicated the receptors, which can be associated with S100A8/A9 proteins on cell membrane of NPC using both bioinformatics and experiment validation. The results indicate that RAGE or TLR4 are potential receptors of S100A8/A9, and the blockade of RAGE or TLR4 could obviously affect S100A8/A9 effects on NPC migration and invasion (Supplementary Figure S2). Taken together, these findings indicated that S100A8/A9 stimulation promotes cell proliferation, migration, and invasion, which might be via the receptors of RAGE or TLR4 on NPC.

### 3.4. S100A8/A9 Stimulation Promotes Migration and Invasion of NPC Cells via the p38 MAPK Pathway

Mitogen-activated protein kinase (MAPK) pathway typically responds to extracellular stimulation and is involved into cancer metastasis. S100A8/A9 promote migration and invasion of gastric cancer through the p38 MAPK pathway [31]. To gain insight into the mechanism how S100A8/A9 regulates NPC migration and invasion and explore whether the p38 kinase is also involved into this process, a specific p-38 inhibitor SB203580 was used to block the p38 MAPK pathway. The effect of S100A8/A9 on the migration and invasion ability of NPC cells was tested again by transwell experiments. Importantly, the results showed that p38 MAPK pathway inhibition after SB203580 pretreatment significantly reduced the migration and invasion abilities of these NPC cells even directly cultured in the medium containing 1 *μ*g/ml S100A8/A9 (*P* < 0.05 and *P* < 0.01, respectively (Figures 3(a)–3(d))). However, we tested another MAPKs inhibitor AZD6244, which is a potent, selective MEK1/2 inhibitor as controls. The results indicated that AZD6244 treatment (MEK/ERK pathway inhibition) could not diminish the migration and invasion abilities caused by S100A8/A9 stimulation in all the three NPC cell lines (Supplementary Figure S3). These findings suggested that S100A8/S100A9 might promote the migration and invasion of NPC cells at least through the p38 MAPK pathway.

### 3.5. Tumor Invasion and Migration Associated Proteins *β*-Catenin and MMP7 Were Elevated in Clinical NPC Tissues

We previously discovered that S100A8 and S100A9 knockdown could significantly reduce the expressions of matrix metalloproteinases (MMPs) in NPC cancer cells [30]. In the present study, we further explored the downstream of the signaling pathway and evaluated the *β*-catenin and MMP7 expression levels in clinical NPC tissues and chronic pharyngitis (CP) tissues, which are two important proteins in tumor cell invasion and migration. Here, the clinical tissues result indicated that abundant *β*-catenin and MMP7 proteins were expressed in NPC tissues including II, III, and IV clinical stages. In contrast, only a few *β*-catenin and MMP7 proteins existed in the CP tissues (Figures 4(a) and 4(b). The statistically analyzed results showed that the positive staining area percentage (PSAP) of *β*-catenin and MMP7 in 42 cases of NPC tissues was 13.4 (9.23, 18.52) and 19.6 (11.44, 26.75), respectively, which were higher than those of 4.65 (2.57, 7.19) and 0.8 (0.32, 1.95) in 9 cases of CP tissues, with the significant differences (*z* values −3.83 and −4.59, *P* < 0.01, respectively) (Table S4).

Importantly, the positive stained area percentages of *β*-catenin and MMP7 in II, III, or IV stage NPC tissues were both significantly higher than CP tissues (*P* < 0.01, respectively) (Table S4). In further stratified analysis, the positive staining area percentages of *β*-catenin and MMP7 in advanced stage NPC (III stage or IV stage) were significantly higher than those in the early stage NPC (II stage) (*P* < 0.05 and *P* < 0.01, respectively), while the III stage and IV stage were not statistically different (Table S5).

## 4. Discussion

The expression of S100A8/S100A9 and their roles in NPC tissues is still not very clear up till the present moment. Over the past decade, Cheng et al. identified several proteins including S100A8 and S100A9 higher in NPC tissues than in normal nasopharyngeal epithelial tissues (NNET) by mass spectrometry (MS) [32]. Li et al. also independently discovered that the S100A9 protein in NPC was four times higher than that of NNET [33]. Other experiments including Western blot were subsequently carried out to provide more evidences that S100A9 may be a potential biomarker in NPC tissue, and the S100A9 level is markedly related to clinical typing of NPC [34]. However, it is still unclear that the association between these S100A8/A9 proteins and CP, which is the early lesion ahead of NPC, because this disease stage might affect the specificity of these novel NPC biomarkers. Moreover, the molecular mechanism mediated by S100A8/A9 proteins in NPC migration and invasion is also currently not well understood.

In the past study, we discovered serum S100A8/A9 proteins roughly evaluated in NPC patients as the potential biomarkers, which are highly associated with NPC clinical stages. In the present study, we further detected the intracellular and extracellular S100A8/A9 proteins in NPC tissues and CP tissues. Similar results were observed in accordance with previous serum studies. These S100A8/A9 proteins in the intercellular space of NPC tissues and the cytoplasm of tumor cells were significantly higher than those of CP tissues. Meanwhile, we provide more solid evidences extracted from nearly fifty NPC patients that S100A8/A9 levels were closely related to the clinical stages of NPC, and the advanced stages were significantly higher than the early stages in these NPC tissues. The conclusion is supported by these above evidences that the expression level of S100A8/A9 in NPC tissues is dramatically elevated and closely related to the clinical stages.

To date, overexpressed S100A8/S100A9 proteins have already been observed in a variety of cancer types including breast cancer [35, 36], prostate cancer [37, 38], bladder cancer [39, 40], and colon cancer [41, 42]. S100A8/S100A9 proteins play important roles in promoting cancer proliferation and enhancing their metastasis. Our previous study has shown that silencing of endogenous S100A8/A9 could obviously inhibit the migration of NPC cells [30]. It is well known that pathological stimulation of nasopharyngeal tissue, caused by bacterial/viral infection or inflammation, is a risk factor of NPC [43]. The interactions between NPC cancer cells and stromal cells or immune cells including secrete cytokines act important roles in tumorigenesis [44]. Here, we use exogenous S100A8/A9 protein stimulation to mimic the S100A8/A9 infiltrated NPC microenvironment, where the secreted soluble inflammatory factors S100A8/A9 proteins are observed in the intercellular space and tumor cell cytoplasm of these NPC tissues. Interestingly, our results indicated that as low as 0–5 *μ*g/ml concentration of S100A8/A9 proteins has already tended to promote NPC cell proliferation. In addition, the migration and invasion abilities were markedly enhanced by as low as 1 *μ*g/ml S100A8/A9 proteins in a variety of NPC cell lines including the low-differentiated CNE2 as well as the high-differentiated CNE1 and even low metastatic 6-10B. Similarly, S100A8/A9 at a relatively low concentration (≤25 *μ*g/ml) was reported to promote proliferation, migration, and invasion of breast cancer cells [45]. S100A8/A9 proteins as low as 0.4–2 *μ*g/ml were also discovered to promote migration and invasion abilities in one colorectal cancer study [46]. Taken together, it seems clear from present findings that S100A8/A9 protein stimulation could promote proliferation, migration, and invasion of NPC cells at a low concentration level.

In addition, we also investigated whether the intracellular pathway is involved in S100A8/A9-stimulated NPC migration and invasion. Our findings indicated that this process might be involved into the p38 MAPK pathway. When the p38 MAPK pathway was inhibited, the migration and invasion abilities of NPC cells stimulated by S100A8/A9 were diminished. Consistent with the S100A8/A9 overexpression in NPC clinical tissues, the tumor invasion and migration associated proteins *β*-catenin and MMP7 were also elevated in these clinical NPC tissues. Therefore, here we hypothesized that overexpressed S100A8/A9 as the secreted soluble inflammatory factors in tumor microenvironment might enhance the activity/phosphorylation of the p38 MAPK pathway in cancer cells, which subsequently activated the transcriptional factors and elevated the tumor cell invasion and migration protein expression (e.g., MMP7) and finally promoted NPC cell proliferation, migration, and invasion (Figure 5). As is well known, the p38 MAPK pathway is widely involved into cancer growth, development, proliferation, invasion, migration, metastasis, differentiation, and other physiological processes. The abnormal or excessive activation of the MAPK signaling pathway plays important roles in the malignant transformation and evolution of cells. Of note, a similar mechanism was unraveled that activated the p38 MAPK pathway under the stimulation of exogenous S100A8/A9 could enhance cell proliferation in breast cancer [45] or promoted cell migration and invasion in gastric cancer [31]. In addition, clinical tumor metastasis and invasion/migration are mainly dependent on the activities of protein family-matrix metalloproteinases (MMPs), which are involved into the process of Wnt/*β*-catenin and EMT signaling pathway [47]. Recently, S100A8/9 has been reported to play an important role in intimal hyperplasia by promoting cell growth and angiogenesis via RAGE signaling [48]. Araki et al. also illustrated that the receptor for advanced glycation end products (RAGE) is one of the major S100A8/A9 receptors, which results in the activation of NF*κ*B [49]. Moreover, biologic effects of S100A8/9 via both RAGE and TLR4 on hematopoietic stem cells are by excretion of proinflammatory cytokines in the hematological process [50]. Furthermore, S100A8 and S100A9 induced activation of p38 MAPK signaling was blocked by the toll-like receptor 4 (TLR4) inhibitor [51]. All these references were consistent to our present findings. However, there are few information to clarify the difference between the intracellular and extracellular mechanisms regulated by S100A8/A9 proteins. Although, in the present study, we found both intracellular and extracellular S100A8/A9 displayed the cancer promotion roles in NPC, and further mechanism exploration is needed in the future.

## 5. Conclusion

Taken together, our study reveals that S100A8/A9 proteins are highly expressed in NPC tissues, markedly related to NPC clinical stages. Furthermore, S100A8/A9 overexpression in tumor microenvironment could promote NPC migration and invasion via the p38 MAPK signaling pathway and tumor cell invasion and migration protein overexpression (e.g., MMP7). The discovery of secreted soluble inflammatory factors S100A8/A9 as stimulators of NPC migration and invasion as well as better understanding of the S100A8/A9 actions in microenvironment could provide novel clues for NPC diagnosis and therapy.

## Figures and Tables

**Figure 1:** S100A8 and S100A9 expressions in NPC and CP tissues detected by the immunohistochemistry method. (a) Representative images of S100A8 expression (brown-yellow or tan staining) in positive control (a) (human cervical carcinoma tissue provided by Abcam), CP tissue (b), or NPC tissues in stage II (c), III (d), and IV (e) (magnification 200×). (b) Violin plot of S100A8 positive staining area percentage (PSAP) for CP and NPC tissues including stage II, III, and IV. (c) Representative images of S100A9 expression (brown-yellow or tan staining) in positive control (a) (human spleen tissue provided by Abcam), CP tissue (b), or NPC tissues in stage II (c), III (d), and IV (e) (magnification 200×). (d) Violin plot of S100A8 positive staining area percentage (PSAP) for CP and NPC tissues including stages II, III, and IV. CP, chronic pharyngitis; NPC, nasopharyngeal carcinoma.

**Figure 2:** Effects of exogenous S100A8/A9 stimulation on the cell migration and invasion of NPC cells including CNE1, CNE2, and 6-10B. The lower chamber was filled culture medium with or without S100A8/A9 proteins (1 *μ*g/ml) to explore the migration and invasion abilities of NPC cells including (a) CNE1, (b) CNE2, and (c) 6-10B. The left panels are representative images and right panels are quantifications. *n* = 3, ^*∗∗*^*P* < 0.01.

**Figure 3:** Effects of exogenous S100A8/A9 stimulation on the p38 MAPK pathway in NPC cells. (a) Representative images for the effects of S100A8/A9 proteins on migration of NPC cells after p38 MAPK inhibitor pretreatment (magnification 200×). (b) Quantifications of S100A8/A9 protein effects on migration of NPC cells after p38 MAPK inhibitor pretreatment. *n* = 3, ^*∗∗*^*P* < 0.01. (c) Representative images for the effects of S100A8/A9 proteins on invasion of NPC cells after p38 MAPK inhibitor pretreatment (magnification 200×). (d) Quantifications of S100A8/A9 protein effects on invasion of NPC cells after p38 MAPK inhibitor pretreatment. *n* = 3, ^*∗*^*P* < 0.05 and ^*∗∗*^*P* < 0.01.

**Figure 4:** *β*-Catenin and MMP7 expressions in NPC and CP tissues detected by the immunohistochemistry method. (a) Representative images of *β*-catenin expression (brown-yellow or tan staining) in CP tissue or NPC tissues in stages II, III, and IV (magnification 200×). (b) Representative images of MMP7 expression (brown-yellow or tan staining) in CP tissue or NPC tissues in stages II, III, and IV (magnification 200×). CP, chronic pharyngitis; NPC, nasopharyngeal carcinoma.

**Figure 5:** A hypothesis for the association between SA100A8/A9 proteins and NPC.

## Data Availability

The datasets used and/or analyzed during the current study are available from the corresponding author upon request.

## Abbreviations:

CP: Chronic pharyngitis
iTRAQ: Isobaric tags for relative and absolute quantitation
LC-MS/MS: Liquid chromatography-tandem mass spectrometry
MS: Mass spectrometry
TME: Tumor microenvironment
TI: Tissue infiltration
LNM: Lymph node metastasis
CS: Clinical stage
IHC: Immunohistochemistry
PSAP: Positive staining area percentage
MAPK: Mitogen-activated protein kinase
NNET: Normal nasopharyngeal epithelial tissues.

## Supplementary Materials

Supplementary Materials Supplementary Figure S1. Effects of exogenous S100A8/A9 stimulation on the cell proliferation of NPC cells including CNE1, CNE2, and 6-10B. The cells were treated with S100A8/A9 at different concentrations for 24 hours, respectively. *n* = 9; ^*∗*^*P* < 0.05; ^*∗∗*^*P* < 0.01. Supplementary Figure S2. Effects of exogenous S100A8/A9 stimulation associated with the receptors of both RAGE and TLR4 on NPC cells including CNE1, CNE2, and 6-10B. (a) Bioinformatics prediction indicated both RAGE and TLR4 as the possible receptors of S100A8/A9 stimulation; (b) experimental validation of the possible receptors including RAGE (pretreatment with 50 nM inhibitor FPS-ZM1 for 1 h) and TLR4 (pretreatment with 1 ug/100 ul antibody blocking for 1 h) of S100A8/A9 stimulation on NPC cells. Supplementary Figure S3. Effects of exogenous S100A8/A9 stimulation on another MAPK pathway (MEK1/2) in NPC cells. (a) Representative images for the effects of S100A8/A9 proteins on migration of NPC cells after MEK1/2 inhibitor (AZD6244) pretreatment; (b) quantifications of S100A8/A9 protein effects on migration of NPC cells after MEK1/2 inhibitor (AZD6244) pretreatment. *n* = 3; n.s., not significant; (c) representative images for the effects of S100A8/A9 proteins on invasion of NPC cells after MEK1/2 inhibitor (AZD6244) pretreatment; (d) quantifications of S100A8/A9 protein effects on invasion of NPC cells after MEK1/2 inhibitor (AZD6244) pretreatment. *n* = 3; n.s., not significant. Table S1. Comparison of positive staining area percentage (PSAP) of S100A8 and S100A9 in NPC and CP tissues. Table S2. Comparison of positive staining area percentage of S100A8 and S100A9 in NPC at different clinical stages and CP tissues. Table S3. Correlation between positive staining area percentage of S100A8 and S100A9 in NPC tissues and clinical features. Table S4. Comparison of positive staining area percentage (PSAP) of *β*-catenin and MMP7 in NPC and CP tissues. Table S5. Comparison of positive staining area percentage of *β*-catenin and MMP7 in NPC at different clinical stages and CP tissues

## References

[1] Sham J. S. T., Choy D., Wei W. I. (1990). Detection of subclinical riasopharyngeal carcinoma by fibreoptic endoscopy and multiple biopsy. *The Lancet*.

[2] Corry J., Fisher R., Rischin D., Peters L. J. (2006). Relapse patterns in WHO 2/3 nasopharyngeal cancer: is there a difference between ethnic Asian vs. non-Asian patients?. *International Journal of Radiation Oncology^∗^Biology^∗^Physics*.

[3] Bray F., Ferlay J., Soerjomataram I., Siegel R. L., Torre L. A., Jemal A. (2018). Global cancer statistics 2018: GLOBOCAN estimates of incidence and mortality worldwide for 36 cancers in 185 countries. *CA: A Cancer Journal for Clinicians*.

[4] Yang X., Mo W., Fang Y. (2018). Up-regulation of Polo-like Kinase 1 in nasopharyngeal carcinoma tissues: a comprehensive investigation based on RNA-sequencing, gene chips, and in-house tissue arrays. *American Journal of Translational Research*.

[5] Jiehe W. C. (2017). *Chinese Cancer Registry Annual Report*.

[6] Wei K. R., Zheng R. S., Zhang S. W., Liang Z. H., Li Z. M., Chen W. Q. (2013). Nasopharyngeal carcinoma incidence and mortality in China. *Chinese Journal of Cancer Research*.

[7] Chua M. L. K., Wee J. T. S., Hui E. P., Chan A. T. C. (2016). Nasopharyngeal carcinoma. *The Lancet*.

[8] Palazzi M., Orlandi E., Bossi P. (2009). Further improvement in outcomes of nasopharyngeal carcinoma with optimized radiotherapy and induction plus concomitant chemotherapy: an update of the Milan experience. *International Journal of Radiation Oncology^∗^Biology^∗^Physics*.

[9] Liu G.-Y., Lv X., Wu Y.-S. (2018). Effect of induction chemotherapy with cisplatin, fluorouracil, with or without taxane on locoregionally advanced nasopharyngeal carcinoma: a retrospective, propensity score-matched analysis. *Cancer Communications*.

[10] Peng H., Chen L., Li W.-F. (2017). Tumor response to neoadjuvant chemotherapy predicts long-term survival outcomes in patients with locoregionally advanced nasopharyngeal carcinoma: a secondary analysis of a randomized phase 3 clinical trial. *Cancer*.

[11] Sun P.-Y., Chen Y.-H., Feng X.-B., Yang C.-X., Wu F., Wang R.-S. (2018). High-dose static and dynamic intensity-modulated radiotherapy combined with chemotherapy for patients with locally advanced nasopharyngeal carcinoma improves survival and reduces brainstem toxicity. *Medical Science Monitor*.

[12] Yao J. J., Jin Y. N., Wang S. Y. (2018). The detrimental effects of radiotherapy interruption on local control after concurrent chemoradiotherapy for advanced T-stage nasopharyngeal carcinoma: an observational, prospective analysis. *BMC Cancer*.

[13] Setakornnukul J., Thephamongkhol K. (2018). Neoadjuvant chemotherapy followed by concurrent chemoradiotherapy versus concurrent chemoradiotherapy followed by adjuvant chemotherapy in locally advanced nasopharyngeal carcinoma. *BMC Cancer*.

[14] Liu Y. C., Wang W. Y., Twu C. W. (2018). Comparison long-term outcome of definitive radiotherapy plus different chemotherapy schedules in patients with advanced nasopharyngeal carcinoma. *Scientific Reports*.

[15] Li Y., Chen Q.-Y., Tang L.-Q. (2017). Concurrent chemoradiotherapy with or without cetuximab for stage II to IVb nasopharyngeal carcinoma: a case-control study. *BMC Cancer*.

[16] Gou X. X., Jin F., Wu W. L. (2018). Induction chronomodulated chemotherapy plus radiotherapy for nasopharyngeal carcinoma: a Phase II prospective randomized study. *Journal of Cancer Research and Therapeutics*.

[17] Peng P. J., Lv B. J., Tang C. (2015). Phase II trial of docetaxel combined with nedaplatin for patients with recurrent and metastatic nasopharyngeal carcinoma. *Drug Design, Development and Therapy*.

[18] Wang Y., Wang Z. Q., Jiang Y. X. (2016). A triplet chemotherapy regimen of cisplatin, fluorouracil and paclitaxel for locoregionally recurrent nasopharyngeal carcinoma cases contraindicated for re-irradiation/surgery. *Expert Opinion on Pharmacotherapy*.

[19] Gao Y., Huang H. Q., Bai B., Cai Q. C., Wang X. X., Cai Q. Q. (2014). Treatment outcome of docetaxel, capecitabine and cisplatin regimen for patients with refractory and relapsed nasopharyngeal carcinoma who failed previous platinum-based chemotherapy. *Expert Opinion on Pharmacotherapy*.

[20] Huang Y. J., Xuan C., Zhang B. B. (2009). SELDI-TOF MS profiling of serum for detection of nasopharyngeal carcinoma. *Journal of Experimental & Clinical Cancer Research*.

[21] Han R. R., Huang Y. J., Chen L. (2014). Determination of S100A8 and S100A9 protein in plasma of nasopharyngeal carcinoma patients and its clinical significance. *Chinese Journal of Clinical Laboratory Science*.

[22] Korndörfer I. P., Brueckner F., Skerra A. (2007). The crystal structure of the human (S100A8/S100A9)2 heterotetramer, calprotectin, illustrates how conformational changes of interacting *α*-helices can determine specific association of two EF-hand proteins. *Journal of Molecular Biology*.

[23] Pruenster M., Vogl T., Roth J., Sperandio M. (2016). S100A8/A9: from basic science to clinical application. *Pharmacology & Therapeutics*.

[24] Sleeman J. P. (2012). The metastatic niche and stromal progression. *Cancer Metastasis Reviews*.

[25] Nedjadi T., Evans A., Sheikh A. (2018). S100A8 and S100A9 proteins form part of a paracrine feedback loop between pancreatic cancer cells and monocytes. *BMC Cancer*.

[26] Guo Y., Ji X., Liu J. (2019). Effects of exosomes on pre-metastatic niche formation in tumors. *Molecular Cancer*.

[27] Eisenblaetter M., Flores-Borja F., Lee J. J. (2017). Visualization of tumor-immune interaction - target-specific imaging of S100A8/A9 reveals pre-metastatic niche establishment. *Theranostics*.

[28] Deguchi A., Tomita T., Ohto U. (2016). Eritoran inhibits S100A8-mediated TLR4/MD-2 activation and tumor growth by changing the immune microenvironment. *Oncogene*.

[29] Wang S., Song R., Wang Z., Jing Z., Wang S., Ma J. (2018). S100A8/A9 in inflammation. *Frontiers in Immunology*.

[30] Yan L.-L., Huang Y.-J., Yi X. (2015). Effects of silencing S100A8 and S100A9 with small interfering RNA on the migration of CNE1 nasopharyngeal carcinoma cells. *Oncology Letters*.

[31] Kwon C. H., Moon H. J., Park H. J., Choi J. H., Park D. Y. (2013). S100A8 and S100A9 promotes invasion and migration through p38 mitogen-activated protein kinase-dependent NF-*κ*B activation in gastric cancer cells. *Molecules and Cells*.

[32] Cheng A.-L., Huang W.-G., Chen Z.-C. (2008). Identification of novel nasopharyngeal carcinoma biomarkers by laser capture microdissection and proteomic analysis. *Clinical Cancer Research*.

[33] Li M. X., Xiao Z. Q., Chen Y. H. (2010). Proteomic analysis of the stroma-related proteins in nasopharyngeal carcinoma and normal nasopharyngeal epithelial tissues. *Medical Oncology*.

[34] Li M. X., Xiao Z. Q., Liu Y. F. (2009). Quantitative proteomic analysis of differential proteins in the stroma of nasopharyngeal carcinoma and normal nasopharyngeal epithelial tissue. *Journal of Cellular Biochemistry*.

[35] Yin C., Li H., Zhang B. (2016). Erratum to: RAGE-binding S100A8/A9 promotes the migration and invasion of human breast cancer cells through actin polymerization and epithelial-mesenchymal transition. *Breast Cancer Research and Treatment*.

[36] Tanriover G., Eyinc M. B., Aliyev E., Dilmac S., Erin N. (2018). Presence of S100A8/gr1-positive myeloid-derived suppressor cells in primary tumors and visceral organs invaded by breast carcinoma cells. *Clinical Breast Cancer*.

[37] Hermani A., Deservi B., Medunjanin S., Tessier P., Mayer D. (2006). S100A8 and S100A9 activate MAP kinase and NF-*κ*B signaling pathways and trigger translocation of RAGE in human prostate cancer cells. *Experimental Cell Research*.

[38] Grebhardt S., Veltkamp C., Ströbel P., Mayer D. (2012). Hypoxia and HIF-1 increase S100A8 and S100A9 expression in prostate cancer. *International Journal of Cancer*.

[39] Yao R., Lopez-Beltran A., Maclennan G. T., Montironi R., Eble J. N., Cheng L. (2007). Expression of S100 protein family members in the pathogenesis of bladder tumors. *Anticancer Research*.

[40] Ebbing J., Mathia S., Seibert F. S. (2014). Urinary calprotectin: a new diagnostic marker in urothelial carcinoma of the bladder. *World Journal of Urology*.

[41] Moris D., Spartalis E., Angelou A. (2016). The value of calprotectin S100A8/A9 complex as a biomarker in colorectal cancer: a systematic review. *Journal of B.U.ON Official Journal of the Balkan Union of Oncology*.

[42] Ichikawa M., Williams R., Wang L., Vogl T., Srikrishna G. (2011). S100A8/A9 activate key genes and pathways in colon tumor progression. *Molecular Cancer Research*.

[43] Huang Y. J., Zhang B. B., Ma N., Murata M., Tang A. Z., Huang G. W. (2011). Nitrative and oxidative DNA damage as potential survival biomarkers for nasopharyngeal carcinoma. *Medical Oncology*.

[44] Huang S. C. M., Tsao S. W., Tsang C. M. (2018). Interplay of viral infection, host cell factors and tumor microenvironment in the pathogenesis of nasopharyngeal carcinoma. *Cancers*.

[45] Ghavami S., Rashedi I., Dattilo B. M. (2008). S100A8/A9 at low concentration promotes tumor cell growth via RAGE ligation and MAP kinase-dependent pathway. *Journal of Leukocyte Biology*.

[46] Ang C. W., Nedjadi T., Sheikh A. A. (2010). Smad4 loss is associated with fewer S100A8-positive monocytes in colorectal tumors and attenuated response to S100A8 in colorectal and pancreatic cancer cells. *Carcinogenesis*.

[47] Mao X., Jin Y., Feng T. (2020). Ginsenoside Rg3 inhibits the growth of osteosarcoma and attenuates metastasis through the wnt/beta-catenin and EMT signaling pathway. *Evid Based Complement Alternat Med*.

[48] Zhong X., Xie F., Chen L., Liu Z., Wang Q. (2020). S100A8 and S100A9 promote endothelial cell activation through the RAGE‑mediated mammalian target of rapamycin complex 2 pathway. *Molecular Medicine Reports*.

[49] Araki K., Kinoshita R., Tomonobu N. (2021). The heterodimer S100A8/A9 is a potent therapeutic target for idiopathic pulmonary fibrosis. *Journal of Molecular Medicine*.

[50] Mondet J., Chevalier S., Mossuz P. (2021). Pathogenic roles of S100A8 and S100A9 proteins in acute myeloid and lymphoid leukemia: clinical and therapeutic impacts. *Molecules*.

[51] Kim M. J., Im M. A., Lee J. S. (2019). Effect of S100A8 and S100A9 on expressions of cytokine and skin barrier protein in human keratinocytes. *Molecular Medicine Reports*.

